This article has been retracted.

# An Intelligent Mechanism for COVID-19 Emergency Resource Coordination and Follow-Up Response

**DOI:** 10.1155/2022/2005188

**Published:** 2022-06-20

**Authors:** Hongyan Sun, Wei Xu, Yinyun Yu, Guiyang Cai

**Affiliations:** ^1^School of Management, Shenyang University of Technology, Shenyang 110870, China; ^2^School of Management, Jinan University, Guangzhou 510632, China; ^3^Department of Obstetrics and Gynecology, Shengjing Hospital of China Medical University, Shenyang 110020, China

## Abstract

As a serious emergency in 2020, COVID-19 had a great impact on people's lives. In this paper, short-term and long-term response to emergency supplies needs after the outbreak of COVID-19 in a region is studied. Firstly, a comparative study of different regional resource coordination options in the early stages of COVID-19 is conducted using a multiobjective decision-making approach to arrive at the optimal solution. Then, a system dynamics model is established for the follow-up development of the epidemic, to predict the long-term development trend of the epidemic, and to study the urgency of the needs of different materials in different periods. The results show that time and satisfaction are the two most important indicators in the decision-making of the material deployment programme in the early stages of an outbreak. In the long-term control of the epidemic, the number of patients with minor illnesses generally peaks around 20 days, while the number of patients with severe illnesses generally peaks around 40 days, providing a focus for the supply of supplies at different times in the actual development of the epidemic, in order to better and more effectively control the epidemic and reduce inefficient consumption of supplies.

## 1. Introduction

In late 2019, the city of Wuhan, Hubei Province, reported a number of cases of unexplained pneumonia, and it was quickly confirmed to be contagious, later named COVID-19 [1], which has continued to this day. The COVID-19 is characterized by severity, comprehensive impact, wide scope of development, long duration, and great uncertainty. The response to the epidemic, both in the short term of emergency supplies and in the long term of effective control, is very important.

In the area of epidemic supplies, Fu et al. [2] developed a dynamic synergy model to analyze the link between epidemic prevention and control and the supply chain of supplies. Zeng [3] used fuzzy number and credibility theory to establish a model to find the optimal order quantity of emergency supplies under the epidemic situation. Wu et al. [4] developed an optimization model for the distribution of emergency medical supplies at rescue sites and obtained optimized combinations of different modes of transport and different distribution schemes at rescue sites at different periods of time. Considering the psychology of material demanders, Li et al. [5] constructed a multicycle emergency medical material distribution model by taking patient panic into account. He et al. [6] set up an emergency material distribution model with minimizing the comprehensive jealousy value as one of the optimization objectives.

In terms of the long-term development of the epidemic, Lu et al. [7] proposed a two-stage epidemic model with dynamic control strategy to describe its transmission process. Antony Aroul Raj et al. [8] studied the ability of COVID-19 to spread in different environments, both indoors and outdoors. Sun and Zhai [9] introduced indicators through the Wells-Riley model to study the role of social distance and ventilation effects in preventing the spread of the new crown epidemic. Huang et al. [10] established a system dynamics model to study and analyze the evolution and development of the epidemic. Wu et al. [11] developed a time series neural network prediction model to forecast and analyze the cumulative confirmed cases and deaths. Ding et al. [12] built an agent-based urban simulation model of COVID-19, which could simulate and evaluate the control measures and treatment plans.

The above contents have carried out profound studies on epidemic control and material supply, but most of them focus on long-term development and lack of research on emergency material supply in the early stage of epidemic outbreak. This paper divides epidemic management into short-term and long-term parts. For short-term material coordination, this paper applies a multiobjective decision-making method for the selection of solutions. Multiobjective decision-making is the selection of solutions, not necessarily on the basis of seeking the optimum, but can be on the basis of the most satisfactory and is therefore more suitable for application under complex conditions and better able to solve complex problems [13–16]. In terms of long-term response, this paper uses system dynamics methods to establish a simulation evolution system. Simulation evolution can visualise the increase and decrease of variables while predicting the development of events [17, 18].

## 2. Materials and Methods

### 2.1. Short-Term Emergency Material Coordination Model

Nowadays, the psychological state and emotions of people are increasingly taken into account in the management of incidents [19]. In this paper, satisfaction is chosen as the indicator of the psychological state of the person. Because of the rapid spread and long duration of COVID-19, when an outbreak occurs in one area, it often causes outbreaks at different times, in different places, and on different scales in associated areas. Emergency supplies for COVID-19 include survival supplies such as medical suits, medical masks, test kits, respirators, and other medical supplies. In the early stages of an outbreak, there is often a sharp increase in demand for such materials for a short period of time in order to complete large-scale prevention, control, testing, and treatment of the epidemic virus, and these items have certain requirements for the environment in which they are delivered. As well as the maintenance of normal life and protection, such as food, disinfection supplies, etc., such items need to be supplied to the quarantined population, which is often in large demand, but the demand in terms of time is relatively gentle, and the requirements for transportation conditions are relatively low. For short-term emergencies, the study in this paper focuses on the interregional coordination of resources. This approach can maximize the utilization of resources and prevent some of the materials from being depleted to reduce the value of use because they have not been used for a long time. On the other hand, it can well alleviate the urgency of resource demand and thus smoothly wait for subsequent resource resupply. The selection of coordination scheme is considered from both subjective and objective aspects, and four dimensions are established for measurement. Among them, subjectively, the satisfaction of each of the supply and demand sides is taken as the measurement objective, while objectively, the three dimensions of material satisfaction, time, and cost are considered.

As the supplier of emergency supplies in the short term, the epidemic has been controlled to a certain extent and they have a certain material reserve. At this time, they are more sensitive to the gains and losses of the existing materials. Here, the value function of prospect theory is used to describe the supplier's perceived satisfaction with the demand for emergency supplies:

(1) $$\begin{array}{c} v\left(x\right)=\left\{\begin{array}{cc} {\left(d_{i}-x\right)}^{\alpha }, & d_{i}-x\geq 0,\\ -\lambda {\left[-\left(d_{i}-x\right)\right]}^{\beta }, & d_{i}-x<0, \end{array}\right. \end{array}$$

*x* is the quantity of supplies supplied from the place where the epidemic occurred first to the place where the epidemic occurred later. *λ* represents the characteristic that losses have more influence than gains, which takes the value *λ* > 1. *α* and *β* indicate the degree to which the value curve bends in the face of gains and losses, respectively, so the value function curve is steeper at *x*> *d*_*i*_. The supply side demand perception satisfaction curve is depicted in the figure (see Figure 1). When *x* takes on a value of zero, the place where the epidemic occurred first does not supply supplies to the place where the epidemic occurred later. At this time, the satisfaction of the supplier is the highest, and its satisfaction gradually decreases with the increase of *x*. When the value of *x* reaches *d*_*i*_ (*d*_*i*_ ≥ 0), the value of supply side satisfaction drops to 0. When *x* takes a value of *x*> *d*_*i*_, it drops in a steeper curve, showing loss aversion. The size of *d*_*i*_ can reflect the acceptability of resource supply in the place where the epidemic first occurred and reflect the serious situation of the epidemic at this time. The larger *d*_*i*_ is, the better the epidemic control is.

Considering the particularity of the epidemic, the demand side has different kinds of demand for materials. Therefore, in the study of demand side satisfaction, this paper takes into account the influence of different kinds of materials on the psychological satisfaction degree of the population. Let *R*_*t*_ represent the demand side's resource satisfaction situation at time *t*; that is, the demand side receives the material at time *t* and the demand is partially satisfied. Let *a* denote the critical moment when the satisfaction begins to decline when they do not receive the supplies. And *c* represents the level of material demand (see Figure 2).

(2) $$\begin{array}{c} F\left(R_{t}\right)=\left\{\begin{array}{cc} 1-{\left(R_{t}-a\right)}^{f\left(c\right)}, & t>a,\\ 1, & t\leq a, \end{array}\right.\\ f\left(c\right)=\left\{\begin{array}{cc} 1-u^{2}, & 0<f\left(c\right)<1,\\ \frac{1}{u^{2}}, & f\left(c\right)>1, \end{array}\right.\\ c\in \left(0,1\right), \end{array}$$

0<*f* (*c*) < 1: Emergency supplies necessary for survival. *f* (*c*) > 1: Emergency supplies to maintain normal life.

The overall satisfaction is the weighted function of two kinds of material satisfaction.

(3) $$\begin{array}{c} F=0.5F_{1}+0.5F_{2}. \end{array}$$

After constructing the evaluation system for the indicators of the emergency material coordination program, it is necessary to assign weights to the evaluation indicators. The existing methods for determining the weights of indicator attributes can be divided into three categories: subjective assignment method, objective assignment method, and combination of subjective and objective assignment method. This paper applies a combination of subjective and objective methods.

Entropy weight method can be used to objectively weight various indicators of the scheme [20, 21]. Assume that there are *m* emergency material allocation schemes, and each scheme has *n* evaluation indexes. Let *a*_*ij*_ represent the original value of the *j*-th index of the i-th evaluation object.

(1) Index consistency
Different indicators have different properties and expressions, and according to their properties, they can be divided into positive indicators, negative indicators, and moderate indicators. The research in this paper mainly includes positive indicators and negative indicators.
If *r* is a negative index, it can be converted into a positive index by the following formula:
  (4) $$\begin{array}{c} r_{j}^{\prime }=\max r-r_{j}. \end{array}$$
(2) Dimensionless index
This paper applies the extreme value method as a method of dimensionless processing of the indicators of the emergency material coordination program, converting all indicator values into numbers greater than or equal to 0 and less than or equal to 1. Add a minimum unit value to all index values to ensure compliance with operational requirements. The specific formula is as follows:
Formula of positive index processing:
  (5) $$\begin{array}{c} r_{ij}=\frac{a_{ij}-min\left\{a_{j}\right\}}{\max\left\{a_{j}\right\}-\min\left\{a_{j}\right\}}. \end{array}$$
Formula of reverse index processing:
  (6) $$\begin{array}{c} r_{ij}=\frac{\max\left\{a_{j}\right\}-a_{ij}}{\max\left\{a_{j}\right\}-\min\left\{a_{j}\right\}}. \end{array}$$
(3) The proportion of the original value of the *i*-th evaluation object in the *j*-th index is calculated as *p*_*ij*_
  (7) $$\begin{array}{c} p_{ij}=\frac{r_{ij}}{\sum_{i=1}^{m}r_{ij}}. \end{array}$$
(4) Entropy value *e*_*j*_ of the *j*-th index was calculated:
  (8) $$\begin{array}{c} e_{j}=-\frac{1}{\ln\;m}\sum_{i=1}^{m}p_{ij}*\;\ln\;p_{ij}. \end{array}$$
(5) The difference coefficient *g*_*j*_ of the *j*-th index was calculated:
  (9) $$\begin{array}{c} g_{j}=1-e_{j}. \end{array}$$
(6) Calculate the weight *w*_*j*_ of the *j*-th index
  (10) $$\begin{array}{c} w_{j}=\frac{g_{j}}{\sum_{j=1}^{n}g_{j}}. \end{array}$$
(7) Calculate the composite score
  (11) $$\begin{array}{c} S=\sum_{j=1}^{n}w_{j}*p_{ij}. \end{array}$$

And then, based on the experts' scores, a “0–4 scoring method” can be used to assign subjective weighting to each indicator of the plan. Finally, weight the results of the subjective and objective scoring.

### 2.2. Simulation Modeling of System Dynamics Evolution of COVID-19

The simulation evolution system of COVID-19 established in this paper includes the following decision factors: the coefficient of infection, the times of close contact with the sick person, the vaccination situation, etc. The selection of the above variables for predictive analysis can provide reference for forecasting the demand of different kinds of materials while visually displaying the development status of the epidemic.

Hypothesis of the model:

1. Assume that all infected persons will develop disease, disregarding asymptomatic infected persons.
2. Assume that all patients with severe COVID-19 are converted from mild disease.
3. It is assumed that all COVID-19 involved in the model are transmitted from human to human, and the imported cases are no longer considered after the evolution began.

By studying the transmission mechanism of COVID-19, a feedback diagram of the COVID-19 transmission process can be obtained (see Figure 3).

The feedback graph mainly consists of two loops. The first is a feedback loop consisting of three variables: infection rate, latent patients, and close contacts. They form a positive feedback loop in which the values reinforce each other, making the epidemic worse and worse. The second is a feedback loop composed of five variables: infection rate, latent patients, confirmed rate, confirmed quarantined person, and close contacts. Since the number of negative causal chains is odd, it forms a negative feedback loop, and the interaction between the data enables the epidemic to be alleviated.

Based on this, combined with the further understanding and analysis of COVID-19 epidemic situation, the dynamic flow diagram of COVID-19 can be established (see Figure 4).

The system dynamics flow diagram of COVID-19 epidemic situation established in this paper contains the following variables (see Table 1).

In this paper, the system dynamics software Vensim was used to establish the evolution model, and the values of various variables in the system are assigned by studying the existing official public data and relevant assumptions.

The relationships and functional equations for each variable are shown in Table 2.

## 3. Results

### 3.1. Programme for the Coordination of Short-Term Emergency Supplies

An evaluation index system for coordination of emergency supplies has been established, including 8 indexes in 4 categories (see Table 3).

Four programs *A*–*D* of emergency material coordination were analyzed and the evaluation index values were calculated. The results obtained were shown in Table 4. *X*1–*X*8, respectively, represent the 8 indexes of the evaluation index system of emergency materials coordination program.

First, the indicators of the emergency materials coordination program were standardized (see Table 5).

Entropy weight method was used to calculate entropy weight and entropy value (see Table 6).

The final combined score was calculated as shown in Table 7.

As can be seen from the above table, the final results of the evaluation of the emergency material coordination program indicators, after objective weighting, showed that the priority of the program is *A* > *D* > *B* > *C*, with program *A* being the best.

According to experts' scores, “0–4 scoring method” could be used to subjectively empower various indicators of the plan [22]. In the choice of different schemes, paying attention to different factors will lead to different results. Firstly, the indexes in the scheme were integrated and the average score was obtained (see Table 8).

As can be seen from the above table, the response time is the most important in the selection of emergency supplies coordination plan for the occurrence of an epidemic. The second is the material satisfaction of both sides of the supply and the demand. In addition, the perceived satisfaction of supply and demand is also important. And attention should be paid to reducing the transportation time and cost of materials. The four plans can be ranked and scored according to the order of each index in the table above (see Table 9).

Multiply the index scores of each scheme in Table 9 with the functional importance coefficients in Table 8. The results were shown in Table 10.

The final results of the evaluation of the emergency material coordination program indicators, obtained through the subjective weighting method, showed that the priority of the program was *D*> *A* > *B* > *C*, with program D being the best.

Weight the results of the subjective and objective scoring above (see Tables 7 and 10).

(12) $$\begin{array}{c} P=0.4P_{1}+0.6P_{2}. \end{array}$$

The final results were shown in Table 11.

The comprehensive score of *D* was the highest; that is, Plan *D* was the optimal plan. When the epidemic outbreak occurs, emergency supplies can be coordinated according to Plan *D* in the short term.

### 3.2. Analysis of Simulated Evolutionary Images of COVID-19

In the early stages of COVID-19, the number of cases rises exponentially due to a lack of preparedness. With the number of “mildly ill” patients peaking around 20 days into the outbreak, the demand for medical supplies for the treatment of mildly ill patients is at its peak. Later, as the epidemic is brought under control and the number of people treated falls sharply, the number of mildly ill people can return to its initial state after two months, and after three months it is nearly zero (see Figure 5).

And some patients with mild disease become severe. Under the condition of good treatment, the number of people who become seriously ill is relatively small and will peak around 40 days after the outbreak of the epidemic, when the need for medical supplies for severe cases increases sharply. After that, the number of patients with severe illness drops sharply. In contrast, it takes longer for patients with severe illness to heal. Therefore, the time needed to clear the number of patients with severe illness is much longer than three months, which requires longer follow-up treatment (see Figure 6).

After the outbreak, the number of close contacts of COVID-19 patients changes as shown in the figure (see Figure 7). In the early stage of the outbreak, due to the lack of control of the epidemic, the number of patients in close contact increases sharply. With the discovery and control of the epidemic, the rate of increase in the number of patients in close contact gradually slows down. By 40 days after the outbreak of the epidemic, the rate of increase gradually turns to zero. It can provide reference for the supply of materials such as testing and quarantine of close contacts in the outbreak area.

The change in the number of people cured of COVID-19 is shown in the figure (see Figure 8). In the early days of the epidemic, fewer cases are confirmed, so the number of people cured rose relatively slowly. When a large outbreak occurs, the number of people diagnosed increases rapidly, the number of people treated in isolation increases rapidly, and therefore the number of people cured increases dramatically. The highest rate of cure occurs between 20 and 60 days after the outbreak. And the subsequent epidemic is well controlled, and the number of new cases decreases continuously; that is, the rate of cured people slows down continuously.

## 4. Discussion

The aim of this paper was to study the short-term material coordination and long-term outbreak control after the outbreak of COVID-19 from the perspective of material supply. This paper presented a simulation study of the evolution of COVID-19 under different conditions.

The first was to predict the change in the number of seriously ill patients and deaths under different vaccination states by changing the proportion of the population vaccinated. The graphs (see Figures 9 and 10) show the change in the number of serious illnesses and deaths when the proportion of vaccinated people is 80% and 90%, respectively. It can be seen that increasing the proportion of vaccination can effectively reduce the number of severe patients and deaths; that is, increasing the amount of vaccination can effectively slow down the outbreak and deterioration of the disease.

By changing the variable of isolation intensity, this paper studies the epidemic development under different isolation intensity. The intensity of isolation directly affects the number of people close to the sick. Therefore, we conducted a simulation to analyze the number of close contacts. As shown (see Figure 11), the blue line corresponds to the number of close contacts at a slightly reduced value of isolation intensity. It can be seen that a slight change in isolation intensity will lead to a significant difference in the number of close contacts, and the weakening of isolation intensity will greatly increase the number of close contacts. The increase in the number of people in close proximity means an increase in the number of potentially sick people, which can cause significant problems in the detection and control of COVID-19. Therefore, the timely and rapid isolation of people involved is essential for the effective control of COVID-19 as it develops.

In this paper's study on the coordination of emergency supplies in the short term, the results showed that two factors, time and satisfaction, were critical to the selection of a supplies programme. Time has always been a primary consideration for scholars in the study of emergency supplies deployment. And satisfaction has received increasing attention in recent years [5, 6]. Chen [23] took the limited rationality of human beings into account to build a model of material distribution and used the algorithm to find the optimal solution. Zhu et al. [24] constructed a material dispatching model that took into account the heterogeneous behaviour of disaster victims and decision makers, providing a useful reference for building an efficient emergency relief system.

It is also important to consider the phasing of material requirements. For people in infected areas, the emergency supplies situation will change dynamically over time, and the availability of supplies in the early stages will have a significant impact on the later stages. Li and Su [25] divided the evolution of COVID-19 into four stages: generation, outbreak, peak, and decline, and built a time-varying demand model for medical supplies based on the infectious disease model. Ge and Liu [26] constructed multiple scenarios for the evolution of major infectious diseases in seven dimensions, including time periods, and then addressed the problem of emergency material allocation decisions. This paper applied a system dynamics model to simulate the long-term evolutionary state of COVID-19. Real-time forecasting of the epidemic development was used to understand the subsequent material requirements. COVID-19 are characterized by mutability. However, for the development of the epidemic after mutation, by changing the parameter settings, the research methods of this paper remain applicable.

## 5. Conclusions

As a serious public health emergency, the COVID-19 has an increasingly significant impact on the world. This paper first proposes a method to select a short-term transregional material coordination plan for the epidemic, which can solve the short-term material supply problem. Then, the system dynamics model is used to analyze the long-term development of the epidemic, and a simulation image is obtained. According to the simulation evolution images of different variables, the epidemic development status and the demand for different types of resources can be obtained to provide reference for the subsequent resource supply, so as to achieve the purpose of short-term emergency response and follow-up control of COVID-19. However, the COVID-19 epidemic is still in flux at this stage, and it is only through continuous understanding and research that we can better respond to the epidemic.

## Figures and Tables

**Figure 1:** Function curve of supplier satisfaction. Supply side satisfaction decreases as resource supply increases.

**Figure 2:** Function curve of demand side satisfaction. Demand side satisfaction corresponds to different curves depending on the type of material.

**Figure 3:** Feedback graph. The feedback diagram contains a positive feedback loop and a negative feedback loop.

**Figure 4:** Dynamic flow diagram of COVID-19 transmission. The dynamical flow diagram contains eight state variables, nine rate variables, one auxiliary variable, and 12 constants.

**Figure 5:** Simulation of patients with mild illness. Number of patients with mild illnesses increases and then decreases.

**Figure 6:** Simulation of patients with critical illness. Number of critically ill patients increases and then decreases.

**Figure 7:** Simulation of close contacts. The number of close contacts first increases and then stabilizes.

**Figure 8:** Simulation of healing numbers. The number of cured patients first increases and then gradually stabilizes.

**Figure 9:** Comparison of the number of serious illnesses. The two curves correspond to the changes in the number of critically ill patients at different vaccination rates.

**Figure 10:** Comparison of the number of deaths. The two curves correspond to the changes in the number of deaths at different vaccination rates.

**Figure 11:** Comparison of the number of close contacts. The two curves correspond to the changes in the number of close contacts at different isolation intensities.

**Table 1:** Summary of variables.

Attribute	Name
State variables	Close contacts, vulnerable population, latent patients, diagnosed patients, patients with mild disease, critically ill patients, the number of deaths, the number of cure

Rate variable	Close contact rate, susceptibility rate, infection rates, diagnostic rate, incidence rate, rate of severity, mortality rate, recovery rate 1, recovery rate 2

Instrumental variables	Total number

Constant	Transmission coefficient, contact number, vaccination, coefficient of cure 1, coefficient of cure 2, coefficient of death, *T*1–*T*6

**Table 2:** Relationship and function formula of variables.

formula 1: Close contacts = INTEG (close contact rate)	Formula 7: The number of cure = INTEG (recovery rate 1 + recovery rate 2)	Formula 13: Incidence rate = (Diagnosed patients/*T*2)

Formula 2: Vulnerable population = INTEG (susceptibility rate − infection rates)	Formula 8: The number of deaths = INTEG (mortality rate)	Formula 14: Rate of severe = (0.15 *∗* Patients with mild disease/*T*3 − 0.8*∗*vaccination *∗* 0.15 *∗* patients with mild/*T*3)

Formula 3: Latent patients = INTEG (infection rates − Diagnosed patients)	Formula 9: Close contact rate = (contact number/diagnostic rate)	Formula 15: Recovery rate 1 = (Patients with mild disease*∗*Coefficient of cure 1/T4)

Formula 4: Diagnosed patients = INTEG (diagnostic rate − incidence rate)	Formula 10: Susceptibility rate = (0.5 *∗* Close contacts)	Formula 16: Recovery rate 2 = (critically ill patients*∗*Coefficient of cure 2/T5)

Formula 5: Patients with mild disease = INTEG (incidence rate − recovery rate 1 − rate of severe)	Formula 11: Infection rates = (contact number *∗* Transmission coefficient *∗* vulnerable population *∗* Diagnosed patients/Total number-0.8 *∗* vaccination *∗* Transmission coefficient *∗* Contact number*∗*vulnerable population *∗* Diagnosed patients/Total number)	Formula 17: Mortality rate = (critically ill patients *∗* Coefficient of death/*T*6 − 0.6 *∗* vaccination *∗* critically ill patients/*T*6)

Formula 6: Critically ill patients = INTEG (rate of severe − recovery rate 2 − mortality rate)	Formula 12: Diagnostic rate = (Latent patients/*T*1)	Formula 18: Total number = (The number of cure + vulnerable population + the number of deaths)

Constants: transmission coefficient (*C*1 = 0.24), number of contacts (*C*2 = 8), vaccination (*C*3 = 0.8), coefficient of cure 1 (*C*4 = 0.8), coefficient of cure 2 (*C*5 = 0.6), coefficient of death (*C*6 = 0.15), *T*1–T6. All data are set based on real data.

**Table 3:** Evaluation index system of coordinated program of emergency supplies.

The dimension	Indicators	Symbol	Attribute of a metric
Mutual satisfaction	*Supplier's perceived satisfaction*	*X*1	Positive
	Demander's perceived satisfaction	*X*2	Positive

Material satisfaction	Supply side material satisfaction rate	*X*3	Positive
	Demand side material satisfaction rate	*X*4	Positive

Cost	The cost of transporting materials	*X*5	Negative
	The value cost of material loss	*X*6	Negative

Time	Time for material response	*X*7	Negative
	Transportation time of materials	*X*8	Negative

**Table 4:** Evaluation index values of coordinated programs for emergency supplies.

	*X*1	*X*2	*X*3	*X*4	*X*5	*X*6	*X*7	*X*8
*A*	0.72	0.77	0.7	0.71	22.4	3.7	5.2	9.2
*B*	0.78	0.48	0.75	0.63	20.8	4.6	6.7	14.1
*C*	0.71	0.39	0.73	0.69	25	4.1	7.2	13
*D*	0.67	0.72	0.69	0.74	27.2	3.2	5.7	11.2

**Table 5:** The dimensionless result.

	*X*1	*X*2	*X*3	*X*4	*X*5	*X*6	*X*7	*X*8
*A*	0.4545	1.0000	0.1667	0.7273	0.7500	0.6429	1.0000	1.0000
*B*	1.0000	0.2368	1.0000	0.0000	1.0000	0.0000	0.2500	0.0000
*C*	0.3636	0.0000	0.6667	0.5455	0.3438	0.3571	0.0000	0.2245
*D*	0.0000	0.8684	0.0000	1.0000	0.0000	1.0000	0.7500	0.5918

**Table 6:** Entropy value, coefficient of difference, and weight.

	*X*1	*X*2	*X*3	*X*4	*X*5	*X*6	*X*7	*X*8
Entropy	0.7198	0.6962	0.6615	0.7710	0.7342	0.7354	0.7032	0.6874
Coefficient of difference	0.2802	0.3038	0.3385	0.2290	0.2658	0.2646	0.2968	0.3126
The weight	0.1223	0.1326	0.1477	0.1000	0.1160	0.1155	0.1295	0.1364

**Table 7:** Comprehensive scores.

*A*	0.3575
*B*	0.2344
*C*	0.1587
*D*	0.2494

**Table 8:** Summary of the results of “0–4 scoring method”.

Functional items	*X*1	*X*2	*X*3	*X*4	*X*5	*X*6	*X*7	*X*8	The total score of the function	The importance factor of function	The sorting
*X*1	0	2	2	3	3	3	2	2	17	0.151	4
*X*2	2	0	2	2	3	3	2	2	16	0.143	5
*X*3	2	2	0	2	4	4	2	3	19	0.169	2
*X*4	1	2	2	0	4	4	2	3	18	0.161	3
*X*5	1	1	0	0	0	2	0	1	5	0.045	8
*X*6	1	1	0	0	2	0	0	2	6	0.054	7
*X*7	2	2	2	2	4	4	0	3	19	0.170	1
*X*8	2	2	1	1	3	2	1	0	12	0.107	6
The total									112	1	

**Table 9:** Summary of the scoring results of each scheme.

	*X*1	*X*2	*X*3	*X*4	*X*5	*X*6	*X*7	*X*8	Total score	The sorting
Plan *A*	3	3	2	3	2	2	4	4	20	2
Plan *B*	4	2	4	1	4	1	2	1	15	4
Plan *C*	3	1	4	2	3	3	1	2	16	3
Plan *D*	1	4	2	4	1	4	4	4	23	1

**Table 10:** A summary of the revised scoring results of each scheme.

	*X*1	*X*2	*X*3	*X*4	*X*5	*X*6	*X*7	*X*8	Total score	The sorting
Plan *A*	0.453	0.429	0.338	0.483	0.09	0.108	0.68	0.428	3.009	2
Plan *B*	0.604	0.286	0.676	0.161	0.18	0.054	0.34	0.107	2.408	3
Plan *C*	0.453	0.143	0.676	0.322	0.135	0.162	0.17	0.214	2.275	4
Plan *D*	0.151	0.572	0.338	0.644	0.045	0.216	0.68	0.428	3.074	1

**Table 11:** Comprehensive score of subjective and objective evaluation.

	*A*	*B*	*C*	*D*
Composite scores	3.009	2.408	2.275	3.074

## Data Availability

If required, data can be obtained by contacting the corresponding author, Guiyang Cai, 1259712491@qq.com.
